RETRACTED

# Development and Validation of a Novel Mitophagy-Related Gene Prognostic Signature for Hepatocellular Carcinoma Based on Immunoscore Classification of Tumor

**DOI:** 10.1155/2021/5070099

**Published:** 2021-10-25

**Authors:** Hao Chen, Jinghua Wang, Ruijie Zeng, Yujun Luo, Kehang Guo, Huihuan Wu, Qi Yang, Rui Jiang, Weihong Sha, Zewei Zhuo

**Affiliations:** ^1^Department of Gastroenterology, Guangdong Provincial People's Hospital, Guangdong Academy of Medical Sciences, Guangzhou 510080, China; ^2^Department of Hematology, Guangdong Provincial People's Hospital, Guangdong Academy of Medical Sciences, Guangzhou 510080, China; ^3^Shantou University Medical College, Shantou 515041, China; ^4^School of Medicine, South China University of Technology, Guangzhou 510006, China; ^5^School of Bioscience and Bioengineering, South China University of Technology, Guangzhou 510006, China

## Abstract

Emerging evidence suggested that mitophagy may play an important role in the progression of hepatocellular carcinoma (HCC), whereas the association between mitophagy-related genes and HCC patients' prognosis remains unknown. In this study, we aimed to investigate the potential prognostic values of mitophagy-related genes (MRGs) on HCC patients at the genetic level. According to median immunoscore, we categorized HCC patients from TCGA cohort into two immune score groups, while 39 differential expression MRGs were identified. By using univariate analysis, we screened out 18 survival-associated MRGs, and then, the least absolute shrinkage and selection operator (LASSO) analysis was applied to construct a prognosis model that consisted of 9 MRGs (ATG7, ATG9A, BNIP3L, GABARAPL1, HTRA2, MAP1LC3B2, TFE3, TIGAR, and TOMM70). In our prognostic model, overall survival in the high and low-risk groups was significantly different (*P* < 0.001), and the respective areas under the curve (AUC) of our prognostic model were 0.686 for 3-year survival in the TCGA cohort and 0.776 for 3-year survival in the ICGC cohort. Moreover, we identified the risk score as the independent factor for predicting the HCC patients' prognosis by using single and multifactor analyses, and a nomogram was also constructed for future clinical application. Further functional analyses showed that the immune status between two risk groups was significantly different. Our findings may provide a novel mitophagy-related gene signature, and these will be better used for prognostic prediction in HCC, thus improving patient outcome.

## 1. Introduction

Hepatocellular carcinoma (HCC) is the commonly diagnosed cancer, representing a significant proportion (75–85%) of cases in primary liver cancer. In 2020, approximately 906,000 new cases and 830,000 deaths occur in liver cancer, which has become an increasing threat to human health worldwide [1]. Large heterogeneity of tumor, frequent recurrence, and intrahepatic metastasis led to a poor 5-year survival rate (5-6%) of HCC, making prognostic prediction challenging [2]. Despite some progresses made in HCC treatment, more new therapeutic targets are required to be implemented [3]. Hence, it is of significance to develop a novel biomarker and risk models to forecast HCC patients' prognosis and provide actionable targets for expanding therapeutic options.

RETRACTED

Mitochondria are the dominating power sources of healthy cells. However, they produce lower energy in cancer cells, and the reprograms metabolism is one of the hallmarks of cancer [4]. Mitochondrial autophagy (mitophagy) can remove dysfunctional or unneeded mitochondria by autophagy, which plays an essential process in cellular homeostasis [5]. Recently, mitophagy-related genes (MRGs) such as PINK1, Parkin, FUNDC1, PHB2, and BNIP3 have developed as a potential target for the development of novel therapeutic strategies for overcoming cancer resistance [6]. In 2020, Zhu et al. demonstrated that the abnormal expression of PINK1 can serve well as biomarker for prognosis of patients with HCC by pancancer analysis [7]. Yan et al. identified another novel mitophagy pathway, PHB2-PARL-PGAM5-PINK1 axis, involved in cancer proliferation and progression, which may become a promising target for the anticancer agent [8]. However, such investigations on MRGs are single or small combination studies, and they do not construct a predictive signature for HCC patients. Therefore, a comprehensive study of MRGs on HCC patients' prognosis at the genetic level is urgently needed.

Recently, immunoscore-based tumor classification has reliably estimated the risk and survival outcome in various tumors with improved guidance of diagnosis and prognosis in tumors [9]. Zheng et al. have also reported that immune-based signature can be used for forecasting HCC patients' prognosis, which offers new insight into treatment and prognosis [10]. Despite advances on the association between the immune score and the prognosis of tumor patients, individualized prognostic models using immunoscore-based tumor classification combined with MRGs have been seldomly reported.

Given the significant values of MRGs with a combination of immunoscore-based tumor classification on HCC patients, we developed and validated a novel mitophagy-related gene signature for forecasting HCC patients' prognosis, which may provide new insight into HCC treatment and prognosis.

## 2. Materials and Methods

### 2.1. Data Collection

RNA-sequencing (RNA-seq) information and clinical characteristics of 371 HCC cases were obtained from the TCGA database up to July 21^st^, 2021 (https://portal.gdc.cancer.gov/repository). The RNA-seq and their corresponding clinical information of 243 HCC samples were obtained as a validation cohort from the ICGC portal (https://dcc.icgc.org/projects/LIRI-JP). The immune score of HCC was retrieved from ESTIMATE (https://bioinformatics.mdanderson.org/estimate). 88 MRGs were selected from GeneCards (https://www.genecards.org) based on their relevance score (relevance score >2, Table S1) on July 21, 2021.

RETRACTED

### 2.2. Immunoscore-Based Tumor Classification and Screening Differential MRGs

Using median immune score as the cutoff, 371 HCC cases were categorized into a high immune score group and a low immune score group. 88 MRGs expression profiles were extracted from the TCGA cohort's RNA-seq data, and then, the differentially expressed MRGs were screened out by using the “limma” R package between such two groups with a threshold of *P* < 0.05. Using the “GOplot” package of R, GO enrichment visualization was employed to identify the main biological properties of these differentially expressed MRGs. Protein-protein interaction (PPI) networks of differentially expressed MRGs were obtained from a website called Search Tool for the Retrieval of Interacting Genes (STRING) (https://string-db.org), and the “igraph” package of R was used to analyze the correlation network of these differentially expressed MRGs [11].

### 2.3. Establishment and Verification of the Prognostic Model

Univariate analysis was employed to evaluate overall survival (OS)-related genes, and we performed survival analysis on them. The LASSO algorithm (R package “glmnet”) was further conducted on these OS-related genes to screen out the final gene signature for developing a prognostic model. Penalty parameter (*λ*) for the model was decided by the minimum criteria. Use the “scale” function of R to centralize and normalize the TCGA expression data for calculating the risk score. The formula is given as follows: risk score = sum (corresponding coefficient × each gene's expression level). According to the median value of the risk score, we classified HCC cases into two risk groups (high-risk group and low-risk group). The training set (TCGA cohort) and validation set (ICGC cohort) were both applied to verify the validity of this risk model. Principal component analysis (PCA) was performed by the “prcomp” function in the “stats” R package. Survival analysis was performed to compare the OS time between two risk groups by “survminer” and “survival” packages of R. ROC curve analysis was performed by “survminer,” “survival,” and “time-ROC” of R to evaluate the performance of our prognostic risk score model.

RETRACTED

### 2.4. Estimation of Independent Prognostic Value

HCC patients' clinicopathological characteristics were extracted from the TCGA cohort. The relationship between the clinical variables (age, sex, tumor grade, T stage, N stage, M stage, and tumor stage) and risk model was performed by using univariate and multivariable Cox regression analyses. To better access the role of our risk score in HCC development, we further explore the association between the risk score and HCC patients' clinicopathological characteristics. Subsequently, R packages “rms” and “survival” were applied to develop a nomogram that included each MRG signature in the model to evaluate the role of the prognostic model. The calibration curve and its quantified data of each risk group were performed using the “riskRegression” and “survival” package.

### 2.5. Functional Enrichment Analysis

DEGs between two risk groups were screened out by the criteria (|log_2_FC| ≥ 1, FDR < 0.05). The “clusterProfiler” R package was applied to process Gene Ontology (GO) and Kyoto Encyclopedia of Genes and Genomes (KEGG) analyses [12]. The BH method was used to adjust *P* values. The most notably enriched GO terms and KEGG pathways were visualized by “GOplot” package of R. Tumor Immune Estimation Resource (TIMER) database was performed to analyze the relationships between 9 MRGs expression and immune cell infiltration (https://cistrome.shinyapps.io/timer/). Single-sample gene set enrichment analysis (ssGSEA) enrichment score was performed by the “gsva” of R to assess the link between the immune activity and risk score.

### 2.6. Statistical Analysis

R (version 4.1.0) was used for all statistical analyses. Student's *t*-test was employed to compare gene expression between high and low immune score groups. A log-rank test was applied to compare the OS between two risk groups. The independent predictors of OS were identified by implementing univariate and multivariate Cox regression analyses, while the categorical variables were compared by the chi-squared test. The BH method was used for *P* values adjusting. The Mann–Whitney test was applied to compare the ssGSEA enrichment scores between groups.

## 3. Results

### 3.1. Immune Score of HCC Samples and HCC Patients' Baseline Information

We categorized the RNA expression data of HCC patients from the TCGA database (*n* = 371) into a high immune score group and low immune score group based on the median immune score, preparing for further screening differential genes. The immune score of each sample is given in Table S2. After excluding 6 tumor samples with missing data (follow up with 0 day), 365 HCC samples from the TCGA dataset were included as a training set. The validation set consisted of 243 HCC samples from the ICGC dataset (Table S3).

RETRACTED

### 3.2. Identification of DEGs between High and Low Immune Score Groups

We presented a heatmap of normalized gene expression profiles of 88 MRGs between the high immune score group (*n* = 186) and low immune score group (*n* = 185) (Figure 1(a)). 39 MRGs were differentially expressed between two groups (FDR < 0.05).  Figure 1(b) shows a boxplot of 39 MRGs expression between two immune score groups. GO enrichment analysis showed that these genes were mainly enriched in macroautophagy, autophagosome, mitochondrion, autophagosome membrane, and mitophagy, indicating their tight relationship with mitophagy (Figure 1(c)).  Figure 1(d) shows the correlation network of the mitophagy-related DEGs between two immune score groups, and the colors intensity marked the degree of the relevance. Protein-protein interaction (PPI) analysis was performed to further explore the interactions of these mitophagy-related DEGs (interaction score = 0.700, high confidence). As shown in Figure 1(e), we could find that MAP1LC3A, MAP1LC3B, GABARAP, GABARAPL1, ATG7, ATG14, ATG9A, BNIP3, BNIP3L, OPTN, NBR1, TOMM20, PARK2, and TP53 were hub genes.

### 3.3. Establishment of the Prognostic Risk Model Based on MRG Signature

18 MRGs were associated with patients' survival after using univariate analysis (*P* < 0.05, Figure 2(a)). To further assess the influence of these genes on the survival of HCC patients, we performed survival analyses and found that 9 MRGs (TFE3, PHB, HIF1A, TOMM70, HTRA2, ATG7, TIGAR, ATG9A, and MAP1LC3B2) were correlated with a poor prognosis (all adjusted *P* < 0.05, Figures 2(c)–2(k)), whereas GABAPAPL1 was reversed (adjusted *P* < 0.05, Figure 2(b)). This well illustrated that using immunoscore-based tumor classification can be used to screen out most differentially expressed MRGs with a better survival and prognostic value, which laid a good foundation for developing a prognostic risk model. After LASSO regression analysis of these genes mentioned above, we obtained a 9-gene signature (ATG7, ATG9A, BNIP3L, GABARAPL1, HTRA2, MAP1LC3B2, TFE3, TIGAR, and TOMM70) based on the optimal value of *λ* (0.02719766) (Figures 3(a) and 3(b)). The multivariate Cox regression analysis of these 9 genes confirmed that GABARAPL1, HTRA2, and TOMM70 had significant prognostic values for patients with HCC from the TCGA cohort (*P* < 0.05, Figure 3(c)). The risk score model was established as follows: risk score = (0.345957*∗*MAP1LC3B2+0.145250*∗*TIGAR+0.126953*∗*HTRA2+0.034558*∗*TOMM70+0.034531*∗*ATG9A+0.020504*∗*BNIP3L+0.002834*∗*ATG7+0.000903*∗*TFE3 − 0.014023*∗*GABARAPL1).

RETRACTED

To offer a quantitative method to predict the survival rate of HCC patients, we developed a nomogram according to the risk score and 9-gene signature. The total nomogram score was calculated to predict HCC patients' survival time at 1, 3, and 5 years (Figure 3(d)). The point of each gene was obtained via drawing a line straight upward from each gene to the point scale in the nomogram. Sum each point to the total points and then locate them in the total points scale to further convert to survival probability. The results indicated that the nomogram-predicted risk generally coincided with the estimated actual risk (Figure 3(e)). Quantitation data of the calibration curve has also shown that these values of predicted risk were close to that of the values of estimated actual risk in each risk group (Figure 3(f)). This suggested that our signature-based nomogram could provide a high value to predict the prognosis of HCC patients. According to the median risk score, we classified the HCC cases into a high-risk group (*n* = 182) and a low-risk group (*n* = 183) (Figure 4(a)).  Figure 4(b) shows that the patients in the low-risk group possessed longer survival times and fewer deaths than in the high-risk group. PCA plot demonstrated that patients can be well separated into two clusters according to the risk score (Figure 4(c)). The survival time of the low-risk group was notably better than that of the high-risk group (*P* < 0.001, Figure 4(d)). In addition, to test the reliability of the prognostic model, we performed ROC analysis. As shown in Figure 4(e), the area under the ROC curve (AUC) was 0.743 for 1-year, 0.686 for 3-year, and 0.684 for 5-year survival, indicating that MRGs could be used as a predictor in the prognosis of HCC. Furthermore, a heatmap of the 9-gene signature was drawn between two risk groups in combination with clinical features from the TCGA cohort (Figure 4(f)). We could find that 8 genes (ATG7, ATG9A, BNIP3L, HTRA2, MAP1LC3B2, TFE3, TIGAR, and TOMM70) were upregulated in the high-risk group except for GABARAPL1 (*P* < 0.05).

### 3.4. Validation of the Prognostic Risk Model by the Training Set

We used the external dataset (ICGC cohort) to assess the reliability of the risk model established by 9-gene signature. The multivariate Cox regression analysis of these 9 genes identified that ATG7, HTRA2, and MAP1LC3B2 had significant prognostic values for patients with HCC from the ICGC cohort (*P* < 0.05, Figure 5(a)). Based on the median risk score obtained from the TCGA cohort, we classified the patients from the ICGC cohort into a high-risk group (*n* = 121) and a low-risk group (*n* = 122) (Figure 4(g)). Similar to the results of the previous TCGA cohort, shorter survival times and more deaths occurred in the high-risk group compared to the low-risk group (Figure 4(h)). As expected, PCA plot demonstrated that HCC patients can be well separated into two clusters according to the risk score (Figure 4(i)). Likewise, compared to the high-risk group, the low-risk group showed a better survival (*P* < 0.001, Figure 4(j)). Moreover, the area under the ROC curve was 0.733 for 1-year, 0.769 for 2-year, and 0.776 for 3-year survival (Figure 4(k)), implying that 9-gene signature could be used to predict HCC patients' prognosis from the ICGC cohort as well.  Figure 4(l) shows a heatmap of the expression level of 9-gene signature based on the risk score and corresponding clinical features from the ICGC cohort. The expression level of 9 genes between two risk groups was the same as the result of the TCGA cohort.

RETRACTED

### 3.5. Independent Prognostic Analyses of HCC Patients Based on the Risk Score Model

We combined the clinical parameters of patients' age, sex, tumor grade, T stage, N stage, M stage, and tumor stage to assess whether the risk score was the independent prognostic factor. Univariate Cox regression analysis of HCC cases from the TCGA cohort revealed that tumor stage, T stage, M stage, and risk score had a significant influence on patients' prognosis (*P* < 0.05, Figure 6(a)). In the multivariate Cox regression analysis, risk score was the only independent predictor of HCC patients (*P* < 0.05, Figure 6(b)). Results of the ICGC cohort were consistent with the TCGA cohort after univariate and multivariate Cox regression analyses (Figures 5(b) and 5(c)). Subsequently, we observed the association between the risk score and the clinicopathological features of HCC patients in the TCGA cohort. Status (alive vs. dead, *P* < 0.001), T stage (T1 vs. T4, *P*=0.0172), and tumor stage (stage I; vs. stage III, *P* < 0.001) were strongly associated with our risk score (Figure 6(c)). A gradual increase of the probability of progression to the late-stage tumor is observed with the increased risk score indicating that our risk model may function in the progression of HCC.

### 3.6. Functional Analyses based on the Risk Model

DEGs were screened out by our risk model in the TCGA cohort (Table S4) and the ICGC cohort (Table S5). The result of GO enrichment showed that DEGs were mainly enriched in the olfactory receptor activity, G-protein coupled receptor activity, and detection of chemical stimulus involved in sensory perception of smell in the TCGA cohort, whereas DEGs from the ICGC cohort were significantly enriched in aromatase activity, mitotic nuclear division, and anaphase-promoting complex binding (*P* adjust <0.05, Figures 7(a) and 7(c)). In addition, DEGs from both two cohorts were all associated with the extracellular region (*P* adjust <0.05, Figures 7(a) and 7(c)). In KEGG pathway analysis, DEGs were primarily enriched in cell cycle and the retinol metabolism in both cohorts (*P* < 0.05, Figures 7(b) and 7(d)), indicating that DEGs obtained from our risk model were associated with the energy metabolism and cellular homeostasis.

RETRACTED

### 3.7. Relationship between the Risk Score Model and Immune Activity

We analyzed the associations between 9 prognostic genes expression and six immune infiltration cells by the TIMER database. Among the 9 genes, ATG7, ATG9A, BNIP3L, HTRA2, MAP1LC3B2, TFE3, TIGAR, and TOMM70 were significantly correlated with B cell, CD8^+^ T cell, CD4^+^ T cell, macrophage, neutrophil, and dendritic cell infiltrations in HCC, while GABARAPL1 was inversely correlated with these six immune infiltration cells (Figure 8). For the further purposes of exploring the relationship between risk score and immune activity, ssGSEA was used to analyze the infiltration level of 16 immune cells and 13 immune-related pathways. The score of B cells, mast cells, natural killer (NK) cells, and plasmacytoid dendritic cells (pDCs) of the high-risk group were significantly lower compared to the low-risk group in the TCGA cohort, whereas the score of activated dendritic cells (aDCs) and macrophages is reversed (all adjusted *P* < 0.05, Figure 9(a)). Besides, the expression level of cytolytic activity, type I IFN response, and type II IFN response was also hyporesponsive in the high-risk group compared to the low-risk group from the TCGA cohort, while the MHC class I pathway was opposite (all adjusted *P* < 0.05, Figure 9(b)). Likewise, except for the macrophages cell, the score of B cells, CD8^+^ T cells, neutrophils, NK cells, pDCs, T follicular helper (Tfh), and tumor infiltrating lymphocyte (TIL) was also decreased in the high-risk group from the ICGC cohort (all adjusted *P* < 0.05, Figure 9(c)). Additionally, the expression level of antigen-presenting cell (APC) costimulation, cytokine-cytokine receptor (CCR), cytolytic activity, T cell costimulation, type I IFN response, and type II IFN response were all reduced in the high-risk group compared to the low-risk group of the ICGC cohort (all adjusted *P* < 0.05, Figure 9(d)).

## 4. Discussion

Mitophagy accounts for the maintenance of cellular homeostasis and energy metabolism in cancers [13]. Despite efforts in investigating the role of mitophagy in cancer recurrence or acquired resistance anticancer therapeutics [14, 15], the precise effect of mitophagy in predicting HCC patients' prognosis is still unknown. Herein, we combined MRGs with immunoscore-based tumor classification to construct a 9-gene risk signature for HCC. Both the training set (TCGA cohort) and validation set (ICGC cohort) work well to verify our risk model by comparing OS and ROC curve between groups. Our functional analyses showed that the DEGs between two risk groups were primarily enriched in the extracellular region process, cell cycle, and metabolism-related pathways. Further immune activity analysis had indicated that the high-risk group had a generally reduced level of antitumor immune activity.

RETRACTED

The prognostic model proposed in this study was composed of 9 MRGs (ATG7, ATG9A, BNIP3L, GABARAPL1, HTRA2, MAP1LC3B2, TFE3, TIGAR, and TOMM70). Compared with single or small combination study on MRGs, our study performed a comprehensive study on MRGs for HCC prognosis at the genetic level by using whole transcriptome datasets. Previous studies have also established the prognostic model for predicting HCC patients' survival such as m6A methylation-related [16] or ferroptosis-related gene signature [17] by harnessing gene expression profiles. However, these results lack external datasets [16] and thorough investigation of prognostic signature [17]. Compared to traditional subtype (normal groups versus tumor groups), our MRG signature combined the MRGs with the immunoscore tumor classification to select more stable specific prognostic markers, which has a better prognostic value for the clinical diagnosis and prognosis.

To date, mitophagy has not been fully researched. This is because initiation and progression of a tumor is not a series of isolated mitophagy pathways but instead is a complex process coexisting and interacting with multiple modes of cell death. Therefore, we could find that these 9 genes are also associated with mitochondria regulators (BNIP3L, HTRA2, TFE3, TOMM70), autophagy (ATG7, ATG9A, GABARAPL1, and MAP1LC3B2), apoptosis (HTRA2), and antioxidant activity (TIGAR). BCL-2 interacting protein 3 like (BNIP3L), transcription factor E3 (TFE3), and translocase of outer mitochondrial membrane 70 (TOMM70) have been implicated in modulation of mitochondrial function. BNIP3L can directly target mitochondria by binding to Bcl-2 and promote cancer stemness of HCC by glycolysis metabolism reprogramming [18], whereas TFE3 are involved in PINK1 and Parkin-dependent mitophagy and can promote the proliferation of renal cell carcinoma [19]. Translocase of outer mitochondrial membrane 70 (TOMM70) is a key receptor of hydrophobic preproteins for binding to mitochondria, which can induce apoptosis of hepatoma cells [20]. HTRA2 is a nuclear-encoded mitochondrial serine protease that has been shown to have a dual function including regulation of cellular apoptosis and mitochondrial homeostasis [21]. A recent study has revealed that inhibition of HTRA2 releasing from the mitochondrion can suppress HCC cell apoptosis [22]. Autophagy-related 7 (ATG7), autophagy-related protein 9A (ATG9A), gamma-aminobutyric acid receptor-associated protein-like 1 (GABARAPL1), and microtubule-associated proteins 1A/1B light chain 3 beta 2 (MAP1LC3B2) are mainly involved in autophagosome formation, whereas the absence of them can lead to a reduction of mitochondrial clearance [23–26]. TP53-induced glycolysis regulatory phosphatase (TIGAR), also named C12 or f5, has antioxidant activity and can protect cells from metabolic stress-induced cell death. Previous studies indicated that the expressions of BNIP3L, TFE3, TOMM70, HTRA2, ATG7, ATG9A, MAP1LC3B2, and TIGAR are overexpressed in tumor tissues, and the knockout of them can significantly inhibit tumor outgrowth [20, 22, 27–32]. In contrast, GABARAPL1 expressions were downregulated in cancer, and our survival analysis of GABARAPL1 showed that high GABARAPL1 expression had a better survival outcome in HCC. The same trend goes as their correlations with immune cell infiltration. Except for GABARAPL1, the remaining 8 genes were positively correlated with B cell, CD8^+^ T cell, CD4^+^ T cell, macrophage, neutrophil, and dendritic cell infiltrations in HCC by using the TIMER database, which indicated that these mitophagy signature may play a vital role in immune activity.

RETRACTED

We also analyzed the DEGs between two risk groups and found that DEGs were associated with the extracellular region process, cell cycle, and energy metabolism pathways. Moreover, compared to the low-risk group, the contents of B cells, NK cells, and pDCs were relatively minimal in the high-risk group in both two cohorts, indicating a decreased antitumor immune response in HCC patients' high-risk group. Emergent evidence has indicated the significance of mitochondrial dynamics in these immune cells [33]. Immune cells proliferation and activation lead to increased metabolic demands, and thus, the reduction activity of antitumor activity of these cells may be associated with mitophagy dysfunction [34]. How mitophagy exerts its action in the regulation of immune cells' activation in different stages is worth to be further explored. In addition, the expression level of macrophages was significantly increased in the high-risk group compared to the low-risk group in both two cohorts. Increased macrophages are correlated with poor prognosis because of their important function in innate immunity [35]. Moreover, a high-risk score may link to compromised immune function. In this study, the components of immune-related functions such as cytolytic activity, type I IFN response, and type II IFN response were also reduced in the high-risk group in both two cohorts. Thus, unfavorable prognosis in the high-risk group of HCC patients may be related to lower immune infiltration levels.

RETRACTED

There are several limitations of this study as well. Our analytical data are mainly obtained from the public dataset, and it is necessary to search for more prospective clinical data to prove the practicability of our prognostic risk model. In addition, further in vitro and in vivo verifications are required to elucidate the specific role of MRGs on HCC. In the future, we can pay more attention in the exploration of the specific mechanism of MRGs on progression of HCC, which may provide novel opportunities for the treatment of HCC.

## 5. Conclusions

In summary, we found that MRGs were associated with HCC patients' prognosis and used them to develop and validate a valid prognostic risk model based on 9-gene signature. Risk score calculated by 9-gene signature was confirmed as an independent prognosis risk factor in both the TCGA cohort and ICGC cohort. Risk score calculated by 9-gene signature was confirmed as an independent prognosis risk factor in both two cohorts. The result of our study may be of significance to develop novel prognostic biomarkers and actionable targets for expanding therapeutic options of HCC patients.

## Figures and Tables

**Figure 1:** Gene expression and interaction among MRGs. (a) Gene expression profiles of the MRGs based on immunoscore classification. (b) Gene expression of 39 differentially expressed MRGs between two immune score groups. (c) GO analysis of 39 differentially expressed MRGs. (d) Correlation network of 39 differentially expressed MRGs. The strength of the relevant links to the depth of the colors. (e) PPI network encoded by 39 differentially expressed MRGs.

**Figure 2:** Survival analysis of 39 MRGs. (a) A forest plot of prognosis-related mitophagy genes after univariate analysis, and 18 genes were with *P* < 0.05; when the HR > 1, the gene was regarded as a high-risk gene. HR, hazard ratio. (b)–(k) Survival analysis of 10 significantly different genes. High expression of TFE3, PHB, HIF1A, TOMM70, HTRA2, ATG7, TIGAR, ATG9A, and MAP1LC3B2 was correlated with a poor prognosis, whereas GABAPAPL1 was opposite (all *P* < 0.05).

**Figure 3:** Establishment of the prognosis model according to mitophagy-related gene signature in the TCGA cohort. (a) LASSO regression of the 18 mitophagy genes with the prognosis value. (b) Cross-validation for tuning the parameter selection in the LASSO regression. (c) A forest plot of 9 MRGs by multivariate Cox regression, and GABAPAPL1, HTRA2, and TOMM70 were with *P* < 0.05. (d) Nomogram for predicting the survival rate of HCC patients based on 9-gene signature. (e) Calibration curve of a nomogram. (f) Bar graph of predicted risk data and estimated actual risk data in each risk group.

RETRACTED

**Figure 4:** Prognostic risk model in HCC patients from the training set and validation set. Distribution of HCC patients based on the risk score in the training set (a) and validation set (g). Survival time and survival outcomes for each HCC patient in the training set (b) and validation set (h). PCA plot according to the risk score in the training set (c) and validation set (i). Kaplan–Meier curves for the survival of HCC patients between two risk groups in the training set (d) and validation set (j). ROC curves of HCC patients in the training set (e) and validation set (k). Heatmap of the training set (f) and validation set (l).

**Figure 5:** Univariate and multivariate Cox regression analyses of MRGs and clinical paraments in the ICGC cohort. (a) A forest plot of 9 MRGs by multivariate Cox regression, and ATG7, HTRA2, and MAP1LC3B2 were with *P* < 0.05 Univariate (b) and multivariate analyses (c) of clinical paraments in the ICGC cohort.

**Figure 6:** Univariate and multivariate Cox regression analyses for the risk score. (a) Univariate and (b) multivariate analyses for the TCGA cohort. (c) Correlation of the risk score with status, age, sex, grade, T stage, N stage, M stage, and TNM stage of HCC.

**Figure 7:** Functional analyses of DEGs that were screened between the two risk groups. GO enrichment (a) and KEGG pathways (b) in the training set. GO enrichment (c) and KEGG pathways (d) in the validation set.

**Figure 8:** The correlation between 9 MRGs expression and immune cell infiltration using the TIMER database.

**Figure 9:** The association between immune activity and two risk groups. Enrichment score of immune cells (a) and immune-related pathways (b) in the training set. Enrichment score of immune cells (c) and immune-related pathways (d) in the validation set. Red box represents the high-risk group. Green box represents the low-risk group (the below is the same). Adjusted *P* values: ns, not significant; ^*∗*^*P* < 0.05; ^*∗∗*^*P* < 0.01; ^*∗∗∗*^*P* < 0.001.

## Data Availability

The datasets are available in the TCGA database (https://portal.gdc.cancer.gov/repository) and ICGC portal (https://dcc.icgc.org/projects/LIRI-JP).

## Supplementary Materials

Supplementary Materials Supplementary Table S1. MRGs included in analysis. Supplementary Table S2. The immune score of each HCC sample from TCGA cohort. Supplementary Table S3. Clinicopathologic characteristics of HCC patients. Supplementary Table S4. Differentially expressed genes between the risk groups in the TCGA cohort. Supplementary Table S5. Differentially expressed genes between the risk groups in the ICGC cohort.
